# A multivariate causality analysis of CO_2_ emission, electricity consumption, and economic growth: Evidence from Western and Central Africa^☆^

**DOI:** 10.1016/j.heliyon.2023.e12858

**Published:** 2023-01-07

**Authors:** Samuel Asante Gyamerah, Luis Alberiko Gil-Alana

**Affiliations:** a Department of Statistics and Actuarial Science, Kwame Nkrumah University of Science and Technology, Kumasi, Ghana; b Laboratory for Interdisciplinary Statistical Analysis – Kwame Nkrumah University of Science and Technology, Kumasi, Ghana; c Faculty of Economics, University of Navarra, Pamplona, Spain; d Universidad Francisco de Vitoria, Madrid, Spain

**Keywords:** CO_2_ emissions, Africa, Electricity consumption, Economic growth, Vector error correction model

## Abstract

The vector error correction model is used to examine the short- and long-run impacts of electricity consumption and economic growth on CO_2_ emissions in Western and Central Africa from 1970 to 2020. This paper adopted time series vector error correction model (VECM) approach to conduct stationarity test, cointegration test, stability test, and Granger causality test. Cointegration tests are used to examine the long-run impact of electricity consumption and economic growth on CO_2_ emissions. It was revealed that CO_2_ emission, electricity consumption and economic growth are co-integrated. Electricity consumption and economic growth have a significant and positive effect on CO_2_ emission. The study also revealed that the adjustment process is not driven by electricity consumption, and anytime there is a deviation from the long-run equilibrium, economic growth and CO_2_ emission adjust to restore the long-run equilibrium. From the short-run Granger causality, electricity consumption and economic growth do not Granger cause CO_2_ emissions. However, past values of CO_2_ emissions have an effect on the present value of economic growth. Generally, long-run dynamics of electricity consumption and economic growth were established to have a greater impact on CO_2_ emission than the short-run dynamics. Hence, it is important to promote green economic concepts in the area.

## 1 Introduction

Africa's economy continues to be characterized by an increasing growth trajectory in gross domestic product and growing energy consumption. Countries have focused their capacities on improving economic growth with little attention to the associated externalities relating to environmental quality. However, amid an economic boom, there is a likelihood of larger quantities of greenhouse gas (GHG) emissions, which have economic, health, and environmental implications [1–3]. The increased concentration of greenhouse gas effect spawned the heightened pace of global warming, which has become one of the most serious threats to human life, causing about 10% (i.e. 5 million) global deaths annually from extreme hot and cold weather temperatures [4–6]. Since the 1990s, the worldwide community has acknowledged the existence of global warming, arguing that the most efficient approach to address global climate change is to mitigate the amount of greenhouse gas emissions (in particular CO_2_ emission) into the atmosphere. CO_2_, a long-lived climate enforcer (LLCE) is the major contributor to climate change, having both short-term and long-term effects on climate [7,8]. Owing to this, in numerous countries, there have subsequently been calls for policies that seek to gradually reduce carbon emissions.

Additionally, economic development, cannot be made separate from electric power consumption [9]. There have been numerous studies that have found that there is a positive impact of electric power consumption on economic growth in the long and short run [10–12]. Further, an increase in electric power consumption is associated with increased human activities that can lead to environmental quality loss and degradation [9,13]. Both generation and consumption of electricity have been found to contribute significantly to greenhouse gas concentration registering about a quarter in the contribution of overall GHG in the United States alone [9,14]. In Africa, where hydropower contributes to a greater share of electricity generation, the production of power is expected to have low GHG emissions. But, as seen elsewhere in India and China, the hydropower reservoirs and power usage by the people have medium to high GHG emissions due to the heavy utilization of power for industrial, manufacturing and agricultural activities [15,16]. But in Africa where such innovations are less pursued, is this effect of increasing CO_2_ associated with growing demand for electricity and economic growth?

There is a global interest in studies involving the causal relationship between CO_2_ emissions, energy consumption and economic growth as part of achieving the 2015 United Nations Development Programme's (UNDP's) sustainable development Goal 13 [17,18], which is aimed at actions in reducing climate change and its impacts. Electricity conservation measures and renewable electricity generation have been adopted as policy options for managing Africa's electricity deficit in order to reduce environmental quality loss due to electricity consumption and rising CO_2_ emissions while maintaining economic development and growth. Countries with a robust economy usually create an enormous demand for energy. Energy sources such as oil, gas, and electricity are heavily utilized in numerous industries, including manufacturing, transportation, and services. Compared to other forms of energy, electricity is utilized in all sectors. Therefore, electricity consumption is crucial to the growth of the economy. While the usage of electricity (electricity consumption) is seen as a measure of socioeconomic progress [9, 19], many development practitioners are worried about the amount of CO_2_ released by electricity generation and, consequently, its consumption.

Accordingly, having a clear indication of the causality between electricity power consumption, CO_2_ emissions, and economic growth is crucial for policy planning and pursuing green-related projects as well as renewable sources of energy consumption in the area. These studies for instance could afford governments in the area the opportunity to further prioritize economic development projects, thus reducing the negative externality footprint of greenhouse gas emissions projects. Consequently, this research seeks to add to the current body of literature by studying the causal relationship linking electricity consumption, CO_2_ emissions, and economic growth in Western and Central Africa over the period from 1970 to 2020. The study differs from existing literature [2,[20], [21], [22], [23]] on the nexus of energy consumption, CO_2_ emissions, and economic growth as it does not employ oil, coal, gas, or clean energy consumption as a proxy for energy consumption. Instead, this study employs electricity consumption as a proxy for energy consumption to help determine the role of electricity consumption in economic growth and CO_2_ emissions in Western and Central Africa. This study also differs from the studies of [24–26], who studied country-specific cases in Africa on the nexus of electricity consumption, CO_2_ emissions, and economic growth. That is, this current study investigates the nexus between electricity consumption, CO_2_ emissions, and economic growth in the sub-region (Western and Central Africa). Hence, this study is the first of its kind in the literature to examine the multivariate causality analysis of electricity consumption, CO_2_ emissions, and economic growth in Western and Central Africa.

The remainder of the paper is organized as follows: In section 2, we review related literatures on the study; the data and methods employed in the study is presented in section 3; the empirical findings and discussion are given in section 4; and lastly section 5 contains the study's conclusions.

## 2 Literature review

In this section, we present a review of previous studies from three aspects: the nexus between energy consumption (crude oil, natural gas), economic growth, and CO_2_ emission; the nexus between clean energy consumption, economic growth, and CO_2_ emission; and the nexus between electricity consumption (crude oil, natural gas), economic growth, and CO_2_ emission.

### 2.1 The nexus between energy consumption (oil, natural gas, nuclear, coal), economic growth, and CO_2_ emission

A lot of research has been done in the past two decades to study the relationship linking economic growth, energy consumption (crude oil, natural gas), and CO_2_ emissions [20,21,23,[27], [28], [29]]. This is because of the critical role that economic growth and energy consumption play in CO_2_ emissions. There are numerous conflicting ideas about the relationship linking economic growth, energy consumption and CO_2_ emissions, owing to the fact that the relationship between economic growth, energy consumption and CO_2_ emissions have significant policy implications. For example [27,[29], [30], [31]], concluded that a rise in economic growth result in a rise in CO_2_ emissions. In the study of [21], the author concluded that there is a bi-directional causality between CO_2_ emissions and economic growth and there is a causal relationship between energy consumption and CO_2_ emission. However [1,32], claimed that economic growth does not cause a rise in CO_2_ emissions. In majority of these studies, the exact relationship linking economic growth to CO_2_ emissions was found to be bi-directional in causality, thus causing each other reactively. Energy consumption was also found to granger cause economic growth and CO_2_ emissions uni-directionally [30,31]. [33] used the ARDL bounds tests for cointegrating relationships to investigate the causal link between economic growth and two proxies for energy consumption (total energy consumption per capita and electricity consumption per capita) in Tanzania from 1971 to 2006. Their findings indicated evidence of a consistent long-run relationship between economic growth and the two proxies, whereas only unidirectional causality from total energy consumption per capita to economic growth, and a Granger causality from electricity consumption to economic growth [34]. used the autoregressive distributed lag model to investigate the causal relationships between CO_2_ emissions, energy consumption, economic development, and foreign direct investment (FDI) in six Sub-Saharan African countries: Zimbabwe, the Republic of Congo, the Democratic Republic of Congo, South Africa, Kenya, and Zambia. Their findings revealed that the 4 variables used for the study are cointegrated, and that economic development, energy consumption, and FDI Granger cause CO_2_ emissions. According to the authors, a rise in economic growth in most African countries will result in higher CO_2_ emissions. In a recent study [35], studied the link between economic development and CO_2_ emissions in South Africa and found that the two variables had a significant and positive linear relationship.

### 2.2 The nexus between renewable energy consumption, economic growth, and CO_2_ emission

[36] studied the effects of economic growth, renewable energy consumption on CO_2_ emissions for the USA. The results from the Greggory-Hansen cointegration test show that CO_2_ emissions, economic growth, and renewable energy consumption are cointegrated. Further tests using the ARDL model indicate that an increase in renewable energy consumption mitigates environmental degradation. Using the ARDL [37], examined the nexus between renewable energy consumption, CO_2_ emissions, and economic growth in Tunisia. The evidence from the study revealed that, in the long run, all the variables under study are stable. Nevertheless, there was a bidirectional relationship between economic growth and CO_2_ emissions; renewable energy consumption and economic growth; but no relationship between CO_2_ emissions and renewable energy consumption. In a different study [22], used a novel bootstrapped ARDL bounds test with structural breaks to determine the relationship between clean energy consumption, economic growth, and CO_2_ emissions in the G7 countries. The study revealed that there is no cointegration between economic growth, clean energy consumption, and CO_2_ emissions in Canada, France, Italy, the US, and the UK. Owing to the conflicting evidence in the literature [38], employed the ARDL technique to explore the nexus between CO_2_ emissions, renewable energy consumption, and economic growth in Romania. The empirical evidence revealed that there exists cointegration among the variables under study and an uni-directional causality running from renewable energy consumption to economic growth [39]. noted in their study that CO_2_ emissions and renewable energy consumption have no serious effect on economic growth in West Africa.

### 2.3 The nexus between electricity consumption, economic growth, and CO_2_ emission

Sub-Saharan Africa (SSA) has the highest proportion of its people without access to electricity, particularly in rural areas. In light of this problem [24], explored the causal relationship between electricity consumption, industrialization, economic growth, and CO_2_ emissions in Benin using the ARDL approach. Results from the study indicated that in the short run, a 1% increase in electricity consumption increases CO_2_ emissions by 0.56%; and in the long run, a 1% increase in electricity consumption increases CO_2_ emissions by 0.95%. By examining the impact of electricity consumption on economic growth and CO_2_ emissions in the Middle East [40], concluded in their study that CO_2_ emissions and electricity consumption have a long-run relationship with economic growth. The authors also indicated that there is a bi-directional Granger causality between electricity consumption, economic growth, and CO_2_ emissions [41]. examined the asymmetric relationship between electricity consumption, CO_2_ emissions, and economic growth in 15 countries using the nonlinear ARDL technique. The results from the study confirm a nonlinear cointegration between the variables under study in Cameroon, Canada, Zambia, Congo Republic, and the UK. There is also a long-run asymmetric nexus between electricity consumption, CO_2_ emissions, and economic growth in Canada and Cameroon, but a short-run asymmetric effect in the UK and Congo Republic.

As can be observed, most of the studies focus on the causal relationships between energy use (oil, natural gas, nuclear, coal), CO_2_ emissions, and other factors. However, there is scarcity of literature on the nexus of CO_2_ emissions, electric power (electricity) consumption, and GDP in Western and Central Africa. In order to explore the multivariate causation between electricity consumption, GDP, and carbon emissions in Western and Central Africa, this research employs the vector error correction model (VECM).

Other recent studies dealing with similar issues as those examined in this work include [42–44].

## 3 Data and methodology

Using VECM, this study investigates the causal relationship linking CO_2_ emissions, electricity consumption, and economic growth. The aggregated panel data from 1970 to 2020 for the variables were collected from the World Development Indicator website: https://databank.worldbank.org/source/world-development-indicators.

CO_2_ emissions (measured in CO_2_ emissions per capita), Gross domestic product (GDP), and electric power consumption are used as a measure of environmental degradation, economic growth and electricity consumption, respectively. Fig. 1 shows the respective trend of CO_2_ emissions, electricity consumption, and economic growth for the period under study.

**Fig. 1:** Trend of CO_2_ emission, electric power consumption, and gross domestic product.

In the following subsection we describe the methodology used in the paper and that is based on unit roots, cointegration and Vector Error Correction Models. We use this methodology since it is the most relevant one for the analysis of time series and to determine casual relationships.

### 3.1 Econometric model

This study analyses the relationship between CO_2_ emissions, electricity consumption, and economic growth to form a multivariate framework (regression equation) as given in Equation (1). The general model specification is given below,

(1) $${CO}_{2_{t}}=f\left(\;{EPC}_{t},{GDP}_{t}\;\right)\text{,}$$

where ${CO}_{2_{t}},{EPC}_{t}\text{,}$ and ${GDP}_{t}$ denote CO_2_ emissions (metric tonnes), electric power consumption (in kilowatt hour per capita), and gross domestic product (in current United States Dollars) at time t respectively. The general form of the multivariate framework in Equation (1) can be expanded as,

(2) $${CO}_{2_{t}}=\vartheta_{0}+\vartheta_{1}\;{EPC}_{t}+\vartheta_{2}\;{GDP}_{t}+\varepsilon_{t\;.\;}$$

By applying logarithms to Equation (2), we seek to minimize the multicollinearity in the model and also to achieve a more stable data variance. The result is the log linear quadratic form given in Equation 3

$$\log\;{CO}_{2_{t}}=\kappa_{0}+\kappa_{1}\;\log\;{EPC}_{t}+\kappa_{2}\;\log\;{GDP}_{t}+\varepsilon_{t}$$

(3) $$L{CO}_{2_{t}}=\kappa_{0}+\kappa_{1}L{EPC}_{t}+\kappa_{2}L{GDP}_{t}+\varepsilon_{t}$$

where $L{CO}_{2_{t}}$, $L{EPC}_{t}$, and $L{GDP}_{t}$ denote the logarithmic conversion of ${CO}_{2_{t}}$, ${EPC}_{t}$, and ${GDP}_{t}$ respectively. $\kappa_{0}$, $\kappa_{1}$, $\kappa_{2}$ are the parameters to be estimated and $\varepsilon_{t}$ is the error term.

### 3.2 Test of unit root

The presence of unit roots in the variables is established using the Phillips-Perron (PP) ([45]), augmented Dickey-Fuller (ADF, [46]), andd Ng-Perron unit root [47] tests. These tests do not impose an autoregressive structure on the error term. The presence of unit-root is a precondition for the cointegration test of Johansen [48].

### 3.3 Cointegration

In this paper, the Johansen test [48] is used to investigate the existence of cointegration between CO_2_, GDP, and EPC. It is significant to know that in the multidimensional scenario, the Engle-Granger suffers from omitted variable bias. Therefore, in such cases it is more efficient to use the Johansen test of cointegration. The null hypothesis of the Johansen test of cointegration is that, “CO_2_, GDP, and EPC are not cointegrated”. If the critical value is greater than the trace statistic, we can reject the null hypothesis. This implies that “CO_2_, GDP, and EPC are co-integrated”.

### 3.4 Vector error correction model (VECM)

If CO_2_, GDP, and EPC are integrated in the same order, then there is a long-run bivariate relation between the variables and if cointegration is detected between CO_2_, GDP, and EPC, then there is the presence of long-run equilibrium link between the variables. This study uses VECM to estimate the short-run cointegration between CO_2_, GDP, and EPC. A VECM is therefore a constrained vector autoregression that can deal with non-stationary time series of variables that are in a long-run relationship. The specification of VECM incorporates cointegration relations that control the long-run dynamics of the endogenous variable in converging to their cointegration relationships while taking into consideration the short-run adjustment process. Owing to the fact that the departure from long-run equilibrium is continuously rectified through a step-by-step short-run adjustments, the cointegration term is referred to as the error correction term (ECM). To build the trace error correction model (ECM) [49], incorporated cointegration and ECM.

The Granger causality for CO_2_ emission under the vector error correction model for this study is expressed in Equation (4),

(4) $$\left[\begin{array}{c} \Delta L{CO}_{2_{t}}\\ \Delta L{EPC}_{t}\\ \Delta L{GDP}_{t} \end{array}\right]=\left[\begin{array}{c} \kappa_{1}\\ \kappa_{2}\\ \kappa_{3} \end{array}\right]+\sum_{i=1}^{K}\Delta \left[\begin{array}{ccc} a_{11i} & a_{12i} & a_{13i}\\ a_{21i} & a_{22i} & a_{23i}\\ a_{31i} & a_{32i} & a_{33i} \end{array}\right]\left[\begin{array}{c} \Delta L{CO}_{2_{t-i}}\\ \Delta L{EPC}_{t-i}\\ \Delta L{GDP}_{t-i} \end{array}\right]+\left[\begin{array}{c} \beta_{1}\\ \beta_{2}\\ \beta_{3} \end{array}\right]\;\left[{ECT}_{t-1}\right]+\left[\begin{array}{c} \varepsilon_{1}\\ \varepsilon_{2}\\ \varepsilon_{3} \end{array}\right]\text{,}$$

where the difference operator is represented by Δ; the error correction term is represent as ECT; the coefficient of ECT is represented as β; K, the number of lags; and ε is the error term.

## 4 Empirical results

In Table 1, we present the summary statistics of CO_2_, EPC, and GDP. The Shapiro-Wilk (SW) normality test reveals that none of the variables are normally distributed. This deviation from normality is evident from the excess kurtosis obtained for all the variables. The correlation coefficient values in the table indicate a positive relationship between CO_2_, EPC, and GDP. That is, an increase in electricity power consumption increases CO_2_ and an increase in GDP growth increases CO_2_ emission. Likewise, an increase in electricity power consumption increases GDP growth. This is consistent to the study of [12] who noted that in the long and short-run, there is a positive effect of electricity consumption on economic growth in Finland and Portugal. However, the relation between EPC and GDP is the strongest.

**Table 1:** Descriptive statistics of CO_2,_ EPC, and GDP.

Variables	N	Mean	Maximum	Minimum	Std.Dev.	Kurtosis	SWtest	P-Value	CO_2_	EPC	GDP
CO_2_	61	0.4433	0.6483	0.0909	0.1458	0.5367	0.79515	0.0000^a^	1.0000		
EPC	61	125.00	197.36	73.74	37.7099	−0.8754	09264	0.0013^a^	0.5280	1.0000	
GDP	61	1354.9	1837.8	990.4	247.2006	−1.0389	0.9069	0.0002	0.4786	0.7344	1.0000

a Denotes significance at 1%; SWtest and StdDev denotes Shapiro Wilk's test and standard deviation respectively.

### 4.1 Validity and reliability

Relevant concerns over data quality in this study mainly hinge on validity and reliability. Validity is concerned about the accuracy of measure. Computing to find Cronbach's alpha has been the commonly adopted procedure for finding reliability measure. According to Ref. [50], a Cronbach's alpha less than 0.7 is unacceptable. However, Cronbach's alpha that falls between 0.8 and 0.9 is considered as a good measure of reliability, but 0.9 is an excellent measure of reliability. Testing for the validity and reliability of the variable constructs, the study adopted the Cronbach Alpha. In Table 2, the Cronbach alpha (α) value obtained is 0.847 implying that the data tools used for the study are 84.7% reliable and can be used over time. Table 3 shows that the 95% confidence interval is in the range of 0.832–0.927.

**Table 2:** Reliability statistics.

Cronbach's Alpha	Number of Items
0.891	3

**Table 3:** Boostrap 95% Confidence Interval based on 1000 samples.

2.5%	97.5%
0.832	0.927

### 4.1 The unit root test

The results of the unit root tests (ADF and PP) are shown in Table 4. Both tests show that LCO_2_, LEPC, and LGDP are non-stationary at level, but only became stationary and integrated at the first order I(1) after their first differences***.*** This fulfils the fundamental precondition for Johansen cointegration. On the other hand, using the Ng-Perron unit root test, the test statistics for all the variables are far above the critical value and the null of unit root could not be rejected even at a loose significance level of 5%. The Ng-Perron unit root test confirms the test results using the ADF and PP unit root test.

**Table 4:** Augmented Dicker Fuller, Phillips-Perron, and Ng-Perron unit root tests.

Variable	ADF (Level)		ADF (First Diﬀerence)		PP (Level)			PP (First Diﬀerence)		Order of Integration
	TS	P-Value	TS	P-Value	TS		P-Value			
								TS	P-Value	
LCO_2_	−2.7225	0.2826	−6.6344	<0.01*	−5.3762		0.7996	−49.489	<0.01*	I(1)
LEPC	−2.5895	0.3364	−8.5955	<0.01*	−15.08		0.2125	−61.545	<0.01*	I(1)
LGDP	−2.0377	0.5596	−3.5584	0.0443*		−5.3115	0.8035	−32.325	<0.01*	I(1)

Ng-Perron Unit Root Test				
	Mza	MZt	MSB	MPT
CO2	−0.69172	−0.42625	0.61622	21.8746
GDP	2.03372	1.28214	0.63044	37.4916
ELECT	−4.78358	−1.48849	0.31117	5.25159
5% Asymptotic critical value	−8.10000	−1.98000	0.23300	3.17000

* denotes significance at 5% level; TS represent Test Statistics.

### 4.2 Lag selection for VECM

The application of the Johansen co-integration test is validated by the presence of a similar order of integration, as reported by the ADF and PP unit root tests. However, the optimal lag is determined before estimating the co-integrating among the variables. The choice of an optimal lag is the first step in the Johansen cointegration test. Hence, in this section, the vector autoregression (VAR) specification is used to establish the appropriate lag length for the cointegration test in this section. The results of the VAR lag selection are presented in Table 5. From the table, it is clear that lag 9 has the minimum final prediction error (FPE) and Akaike information criterion (AIC). Consequently, lag 9 (K = 9) is selected as the optimal lag in the equation models.

**Table 5:** Optimal lag selection using VAR.

	1	2	3	4	5	6	7	8	9	10
AIC	−17.687	17.642	17.683	−17.571	−17.449	−17.230	−17.829	−17.842	−18.126	−18.036
HQ	−17.514	−17.338	−17.249	−17.006	−16.754	−16.405	−16.874	−16.756	−16.910	−16.689
FPE	2.0839e-08	2.1893e-08	2.123085e-08	2.4215e-08	2.8220e-08	3.6831e-08	2.1658e-08	2.3523e-08	2.0187e-08	2.6406e-08

### 4.3 Cointegration test

Before testing for cointegration, two different competing models (Restricted Trend and Intercept Case) of the Johansen cointegration test are compared. The model with the lowest AIC and BIC and the largest log-likelihood is selected as the optimal model for the cointegration test. Table 6 shows the results from the two models. The restricted trend case has lower AIC and BIC values and a larger log-likelihood value. A further test using the likelihood ratio test confirms that the null hypothesis of no inclusion of a linear trend in a VAR can be rejected at a 5% level of significance. Hence, the model from the restricted trend case is selected as the final VEC model. We can therefore conclude that LCO_2_, LEPC, and LGDP show a general stochastic trend over the long term.

**Table 6:** Selection of Restricted Trend and Constant Case competing models.

Selection Criteria	Restricted Trend Case	Intercept Case
AIC	**−928.2272**	−927.3644
BIC	**−772.1278**	−771.2649
Log-likelihood	**322.7592**	322.3278
	Test Statistics	P-Value
LR Test	11.8200	0.0000^a^

a Denotes significance at 5%.

Co-integration among the variables under study is explored using the Johansen cointegration test which is presented in Table 7. From the max-eigenvalue and trace test and at 5% significance level, there can only be one cointegrating relationship. Thus, if we decide to describe our data series using the restricted trend case in this study, one cointegration equation should be assumed. Therefore, the study concludes that there is a long run relationship between CO_2_ emissions, electricity consumption, and economic growth in Western and Central Africa.

**Table 7:** Johansen Cointegration test.

Maximum rank	Eigen Value	Trace Statistics			Max-eigen Statistics		5% CV
		Test Statistics	P-Value	5% CV	Max Statistics	P-Value	
0	0.7529	94.5828	<0.001^a^	42.44	72.6952	<0.001^a^	42.44
1	0.2418	21.8875	0.1460	25.32	14.3950	0.2364	25.32
2	0.1134	7.4925	0.3049	12.25	7.4925	0.3054	12.25

a Denotes significance at the 5% level; CV represents critical value.

### 4.4 VECM estimation and analysis

The presence of cointegration relationships between LCO_2_, LEPC, and LGDP suggests a long-run cointegrating relation between CO_2_ emission, electricity consumption, and economic growth. Hence, the VECM can be applied.

Using the maximum likelihood estimator, the cointegrating coefficient vector normalized to LCO_2_ which is the variable of interest is estimated as given in Table 8.

**Table 8:** Cointegration coefficient vector from VECM.

	LCO_2_	LEPC	LGDP	Trend
Coefficient	1	−0.0316	−0.4895	0.0227

The long-run relationship between LCO_2_, LEPC, and LGDP for a co-integrating vector is,

(5) $$L{CO}_{2_{t}}=0.0316L{EPC}_{t}+0.4895L{GDP}_{t}-0.0104t$$

From Equation (5), an increase in LEPC and LGDP is related to an increase in LCO_2_ emissions. That is, a percentage rise in electricity consumption is likely to cause a 0.0316% increase in CO_2_ emissions. CO_2_ emission is projected to increase by 0.4895% for every percentage point increase in economic growth. This indicates that an increase in electricity consumption and economic growth will result in an increase in CO_2_ emission in the long-run. These findings are similar to the studies of [23,28], although they differ from the conclusion of [1].

Table 9 shows the adjustment coefficients of ECT that measures the rate of convergence of short-run in relation to long-run and test for weak exogeneity. Table 9 shows that at a 5% level, LCO_2_ has a negative (−0.4113) but statistically significant error correction term. This indicates that, not only is there a long-run equilibrium relation between the independent (LEPC and LGDP) and dependent (LCO_2_) variables at the 5% level, but its relative value (−0.4113) for Western and Central Africa reflects the rate of convergence to the equilibrium state each year. The presence of a long-run equilibrium relationship running from electric power consumption and GDP to CO_2_ emission is further demonstrated by the negative but statistically significant error correction term. As shown in Table 9, LEPC is not exogenous because at the 5% level, it is not statistically significant. This shows that whenever there is a departure from long-run equilibrium, the other variables (LCO_2_, LGDP) will adjust to restore long-run stability. That is, the adjustment process is not driven by the weakly exogenous variable (LEPC). Specifically, the rate of adjustment of any imbalance in the direction of a long-run balance is that approximately 41.13% of the discrepancy between the real value and the long-run value is adjusted each year.

**Table 9:** Long-run multivariate causality of the error correction model (ECM).

	$\Delta L{CO}_{2_{t}}$	$\Delta L{EPC}_{t}$	$\Delta L{GDP}_{t}$
ECM(-1)	−0.4113 [0.0476]	0.0607 [0.0502]	−0.0870[0.0189]
P-Value	4.0538e-09^a^	0.2376	9.4029e-05^a^

a Denotes significance at 5%.

At the 5% level, the coefficients of the first differences of LEPC and LGDP lagged one year in LCO_2_ are statistically, according to Table 9. This signifies that there is no short-run causality from electric power consumption and GDP to CO_2_ emission based on VECM estimates. To confirm this short-run causality, a Granger causality test is performed.

### 4.5 Test of granger causality

The Johansen cointegration test proves the presence of causation between the variables, but failed to suggest the direction of the causation. It is therefore imperative to examine the causal link between the variables using the Granger causality test [49]. Table 10 is the summary of the multivariate causality derived from Table 9.

**Table 10:** Multivariate causality tests based on VECM.

Q	P		
	LCO_2_	LEPC	LGDP
LCO_2_	–	0.3129	0.1090
LEPC	0.0833	–	0.0006^a^
LGDP	0.0178^a^	0.0098^a^	–

a Denotes rejection of the hypothesis (P does not Granger cause Q) at the 5% significance level.

There is a unidirectional Granger causality from LCO2 to LGDP, as seen in Table 10. This means that, beyond the information contained in the prior values of economic growth alone, prior values of CO_2_ emission can predict the present values of economic growth, but prior values of economic growth cannot predict the present values of CO_2_ emission. However, there is no directional Granger causality between LEPC and LCO_2_.

### 4.6 Diagnostic tests and stability test

The study investigates the robustness of the VECM by investigating the serial correlation, heteroscedasticity, and normality tests in order to make unbiased statistical inferences. To guarantee the fitness of the constructed model, we performed several diagnostic tests (normality, serial correlation, and heteroscedasticity) on the constructed model. Evidence from.

The residuals are clearly not serially correlated and homoscedastic, as seen in Table 11. The residuals are not jointly normally distributed.

**Table 11:** Long-run multivariate causality of the error correction model (ECM).

	$H_{o}$	Chi-Squared	P-Value
Portamanteau test	No serial correlation up to lag K	173.51	0.8267
Heteroscedasticity	Residuals are homoscedastic	258	0.9972
Normality tests	Residuals are multivariate normal	19.7610	0.0031^a^

a Denotes significance at 5%.

### 4.7 Variance decomposition tests

Both the VECM and the linear regression model are unable to take into account arbitrary innovations that influence the variables in the VAR. To trace back shocks into the future, the study uses the Cholesky variance decomposition technique. Evidence from Table 12 demonstrates that 11% and 25% of future shocks in CO_2_ emissions are caused by electricity consumption and economic growth, respectively. 7% and 16% of future shocks in electricity consumption are caused by carbon dioxide emissions and economic growth, respectively. In addition, 3% and 54% of future shocks in economic growth are caused by carbon dioxide emissions and electricity consumption, respectively. It is evident from the variance decomposition findings in Table 12 that 63.32%, 76.87%, and 43.50% portions of CO_2_ emissions, electricity consumption, and economic growth are contributed by their own innovative shocks. Clearly, the percentage contribution of electricity consumption to economic growth in Western and Central Africa is indicative of the critical role of electricity in sustainable economic growth in this region. The analysis also reveals the contribution of electricity consumption and economic growth to carbon dioxide emissions.

**Table 12:** Variance decomposition analysis.

Period	Variance Decomposition LCO_2_		
	LCO_2_	LEPC	LGDP
1	1.0000	0.0000	0.0000
2	0.8800	0.0016	0.1184
3	0.7939	0.0086	0.1974
4	0.7422	0.0168	0.2410
5	0.7067	0.0186	0.2747
6	0.7016	0.0234	0.2749
7	0.6449	0.1015	0.2536
8	0.6378	0.1108	0.2514
9	0.6295	0.1133	0.2571
10	0.6362	0.1111	0.2527
Period	Variance Decomposition LEPC		
	LCO_2_	LEPC	LGDP
1	1.2699e-07	0.9999	0.0000
2	4.2804e-03	0.9503	0.0454
3	6.8989e-03	0.8666	0.1265
4	5.2765e-02	0.7871	0.1601
5	5.3775e-02	0.7866	0.1596
6	5.6114e-02	0.7847	0.1592
7	7.1353e-02	0.7613	0.1674
8	7.4772e-02	0.7584	0.1668
9	7.3796e-02	0.7564	0.1698
10	6.8789e-02	0.7687	0.1626
Period	Variance Decomposition LGDP		
	LCO_2_	LEPC	LGDP
1	0.4604	0.0003	0.5393
2	0.3508	0.0007	0.6485
3	0.2312	0.0276	0.7413
4	0.1538	0.0699	0.7762
5	0.1063	0.1570	0.7367
6	0.0744	0.2399	0.6857
7	0.0514	0.3411	0.6075
8	0.0398	0.4239	0.5363
9	0.0321	0.4925	0.4754
10	0.0268	0.5382	0.4350

## 4.8 Discussion

Generally, from the Granger causality test, past values of electricity consumption and economic growth do not have an effect on the current emission of CO_2_ in Western and Central Africa. This result is in agreement with the previous results achieved from VECM that at 5% level of significance, there is no short-run causality and is consistent with the result of [51]. This result is in contrast to the study of [28] who concluded that economic growth in China does result in CO_2_ emission. This disparity may be a result of industrialization playing a major role in China's economy as compared to agriculture being the backbone of most Western and Central African economies. This can be ascertained from the study of [27]. The authors concluded that beyond basic industrialization, any relationship between GDP and CO_2_ emissions appears to be very weak. A bidirectional causality exists from LGDP to LEPC.

According to the findings, economic growth and electricity consumption in Western and Central Africa do cause environmental degradation because countries in this region, the majority of which are developing countries, use non-renewable energy resources for industrial and other economic activities that increase CO_2_ emissions in society. The results obtained is consistent with the studies of [25,52]. .Similar to the results obtained in this study [52], and posited that there is a between CO_2_ emissions, electricity consumption, economic growth. However, the study differs from the studies of [1,32] who claimed that economic growth does not cause a rise in CO_2_ emissions.

## 5 Conclusion, policy recommendations, and future studies

Using a vector error correction (VECM) model, multivariate causality analysis between CO_2_ emissions, electric power consumption (proxied as electricity consumption), and GDP (proxied as economic growth) in Western and Central Africa is explored in this work.

Generally, the estimation procedure involved four steps: unit root testing using augmented Dicker Fuller and Phillip-Perron; determining the optimal lag length using vector autoregression techniques; cointegration test using Johansen cointegration test; and investigating the short- and long-run nexus between electric power consumption, gross domestic product and CO_2_ emission via Granger causality tests based on a VECM. Additionally, the study performed several diagnostic tests.

In the long-run, the evidence from the VECM shows that CO_2_ emissions, electric power consumption and GDP are cointegrated. There is a unidirectional causality from CO_2_ emission to economic growth, but there is no directional causality between CO_2_ emission and electric power consumption. Statistical tests from the long-run causality reveal that a percentage increase in electric power consumption and GDP is likely to increase the emission of CO_2_ by 0.0812% and 0.4987% respectively in West and Central Africa. This means that in the long-run, an increase in electric power consumption and GDP will increase CO_2_ emissions. Also, there is statistical evidence of the absence of short-run equilibrium from electric power consumption and GDP to CO_2_ emissions.

The following policy recommendations are made based on the study's findings:

• the two regional blocks should promote green economic policies such as green credit, green bonds, green insurance, green securities to curtail the impact of economic growth on CO_2_ emissions.
• Since an increase in electricity consumption increases CO_2_ emissions, the two regional blocks (Western and Central Africa) should advocate for clean and renewable energy sources such as solar and wind as alternative means of electricity production to ensure sustainable growth of the economy.

The results in this work show that the individual series are nonstationary I(1). However, unit root tests have low power if the data are fractionally integrated. Thus, fractional orders of integration can also be taken into account when analyzing these series. By extension, the long run equilibrium relationship can also be examined from a fractional viewpoint, using fractionally cointegrated models or by using the FCVAR approach developed in Refs. [53,54]. Work in these directions is now in progress.

## Ethical approval

N/A

## Consent to participate

N/A

Consent to publish

N/A

## Competing interests

There are no competing interests with the publication of the present manuscript.

## Availability of data and materials

Data are available from the authors upon request.

## Figures and Tables

**Table A1:** VECM estimation results and test

Error Correction	LCO_2_	LEPC	LGDP
CointEq1	−0.4113(0.0476)***	0.0607(0.0502)	−0.0870(0.0189)***
LCO(-1)	0.3108(0.1467)*	−0.2190(0.1547)	−0.0520(0.0581)
LCO(-2)	−0.1025(0.1848)	−0.1168(0.1433)	−0.0707(0.0539)
LCO(-3)	−0.1847(0.1222)	0.2641(0.1288).	−0.0269(0.0484)
LCO(-4)	−0.0939(0.1269)	0.0666(0.1338)	−0.0177(0.0503)
LCO(-5)	−0.0916(0.1115)	−0.0696(0.1175)	−0.0570(0.0442)
LCO(-6)	−0.1152(0.1156)	0.0631(0.1218)	−0.0035(0.0458)
LCO(-7)	0.0635(0.1097)	0.1712(0.1156)	0.1019(0.0435)*
LCO(-8)	−0.0559(0.1233)	0.0749(0.1300)	−0.1037(0.0489)*
LEPC(-1)	−0.1025(0.1848)	−0.2049(0.1948)	−0.0136(0.0732)
LEPC(-2)	−0.2269(0.1741)	−0.3845(0.1836)*	−0.1103(0.0690)
LEPC(-3)	−0.3677(0.1925).	0.1036(0.2030)	−0.1022(0.0763)
LEPC(-4)	−0.1718(0.1913)	−0.1728(0.2016)	−0.2145(0.0758)**
LEPC(-5)	−0.3933(0.2115).	0.1979(0.2229)	−0.1296(0.0838)
LEPC(-6)	0.0977(0.2067)	0.0862(0.2179)	−0.2622(0.0819)**
LEPC(-7)	−0.4880(0.2473).	0.5078(0.2607).	0.0130(0.0980)
LEPC(-8)	−0.0323(0.2199)	0.0857(0.2318)	−0.1270(0.0872)
LGDP(-1)	−1.3347(0.5782)*	1.0530(0.6095).	0.3461(0.2291)
LGDP(-2)	0.4418(0.4771)	0.3239(0.5029)	0.0181(0.1891)
LGDP(-3)	0.2575(0.3636)	0.1445(0.3832)	0.0714(0.1441)
LGDP(-4)	0.0641(0.3551)	−0.5152(0.3743)	0.0204(0.1407)
LGDP(-5)	0.5384(0.3637)	0.3945(0.3834)	0.3756(0.1441)*
LGDP(-6)	0.4236(0.3971)	0.1787(0.4185)	0.1823(0.1574)
LGDP(-7)	−0.5760(0.3893)	−0.5753(0.4104)	−0.4322(0.1543)**
LGDP(-8)	0.7681(0.3849).	−0.2726(0.4058)	0.3634(0.1526)*
C	−5.4004(0.6259)***	0.7819(0.6598)	−1.1263(0.2481)***
Log likelihood			322.7592
AIC			−928.2272
BIC			−772.1278

***, **, *, denotes significance at 0, 0.001, 0.01, and 0.05 respectively.
